The article "RUNX3 Expression Level Is Correlated with the Clinical and Pathological Characteristics in Endometrial Cancer: A Systematic Review and Meta-analysis" was retracted in 2023. Reasons: signs of a paper mill; compromised peer review; unreliable results or conclusions.

# RUNX3 Expression Level Is Correlated with the Clinical and Pathological Characteristics in Endometrial Cancer: A Systematic Review and Meta-analysis

**DOI:** 10.1155/2021/9995384

**Published:** 2021-07-14

**Authors:** Zhen Liu, Zhi-pan Hong, Shu-xue Xi

**Affiliations:** ^1^Department of Gynecology, Chifeng Municipal Hospital, Chifeng Clinical Medical School of Inner Mongolia Medical University, Chifeng, China; ^2^Department of Tumor Surgery, Chifeng Municipal Hospital, Chifeng Clinical Medical School of Inner Mongolia Medical University, Chifeng, China; ^3^Geneis (Beijing) Co. Ltd., Beijing 100102, China; ^4^Qingdao Geneis Institute of Big Data Mining and Precision Medicine, Qingdao 266000, China

## Abstract

Human Runt-associated transcription factor 3 (RUNX3) plays an important role in the development and progression of endometrial cancer (EC). However, the clinical and pathological significance of RUNX3 in EC needs to be further studied. In order to clarify the clinical and pathological significance of RUNX3, a systematic review and meta-analysis was conducted in EC patients. Keywords RUNX3, endometrial cancer, and uterine cancer were searched in Cochrane Library, Web of Knowledge, PubMed, CBM, MEDLINE, and Chinese CNKI database for data up to Dec 31, 2018. References, abstracts, and meeting proceedings were manually searched in supplementary. Outcomes were various clinical and pathological features. The two reviewers performed the literature searching, data extracting, and method assessing independently. Meta-analysis was performed by RevMan5.3.0. A total of 563 EC patients were enrolled from eight studies. Meta-analysis results showed that the expression of RUNX3 has significant differences in these comparisons: lymph node (LN) metastasis vs. non-LN metastasis (*P* = 0.26), EC tissues vs. normal tissues (*P* < 0.00001), clinical stages I/II vs. II/IV (*P* < 0.00001), muscular infiltration < 1/2 vs. muscular infiltration ≥ 1/2 (*P* < 0.00001), and G1 vs. G2/G3 (*P* < 0.00001). The decreasing expression of RUNX3 is associated with poor TNM stage and muscular infiltration. It is indicated that RUNX3 was involved in the suppression effect of EC. However, further multicenter randomized controlled trials are needed considering the small sample size of the included trials.

## 1. Introduction

Endometrial cancer (EC) is a malignant tumour of uterine epithelial cells. EC is common in postmenopausal women over the age of 50, the incidence of which peaks at the age of 50–59. In developed countries, the incidence of EC occupies the first place in gynaecological tumours [1]. EC is a multifactor process in which the deletion of tumour suppressor genes and the activation of carcinogenesis are particularly important [2, 3]. Though there are many studies exploring cancer-associated biomarkers like genes and noncoding RNAs [4–7], the molecular mechanism of EC is largely unknown.

In recent years, the role of human Runt-associated transcription factor 3 (RUNX3) in the development and progression of EC has attracted increasing attention [8]. RUNX3 is located in human chromosome 1p36.11, and its total length is approximately 67 kb [9]. RUNX3 is an important tumour candidate suppressor gene that is closely related to gastric cancer, breast cancer, gallbladder cancer, and other malignant tumours [10–16]. However, despite numerous patients with EC worldwide, RUNX3 in EC has not been definitively reported, especially on the correlation of its overexpression and its clinical significance in endometrial cancer. Here, we performed a systematic literature review and meta-analysis to determine the association between RUNX3 and the clinicopathological characteristics of EC.

## 2. Materials and Methods

### 2.1. Literature Information

A total of 412 articles were initially identified using the below search strategy. Based on titles and abstracts, 378 out of the 412 were excluded due to non-endometrial-related studies, nonoriginal articles (e.g., review and letter), and duplicate studies. After reading the full texts, we excluded 21 data that could not be extracted due to non-RUNX3-related studies, nonimmunohistochemical SP method, and disunited positive criteria. Eventually, 8 studies (2 in English and 6 in Chinese) were included in the meta-analysis (Figure 1) [17–22].

### 2.2. Study Characteristics

The eight studies included were based on the Asian population, 6 of which were conducted in China, 1 in Japan, and 1 in Korea, involving a total of 827 patients. The overall median age ranged at 28–72 years. The total positive rate of low RUNX3 expression by immunohistochemistry (IHC) is 68.07% from eight studies (from 26.4% to 82.7%). All detected specimens were derived from EC tissues by either biopsy or surgical resection and were confirmed by IHC on membrane protein level. The studies were divided into five groups according to the following criteria: (1) low RUNX3 expression in EC tissues or normal endometrial cancer, (2) low RUNX3 expression in positive and negative lymph node (LN) metastasis of EC tissues, (3) low RUNX3 expression in different clinical stages of EC tissues, (4) low RUNX3 expression in different infiltration degree of EC tissues, and (5) low RUNX3 expression in different pathological stages of EC tissues (Table 1).

### 2.3. Literature Search Strategy

The electronic databases Cochrane Library, PubMed, MEDLINE, Web of Knowledge, and Chinese CNKI and CBM were comprehensively searched for data dated up to Dec 31, 2018. The search string of PubMed was (“RUNX3” [Title/Abstract]) OR “RUNT” [Title/Abstract] AND (uterus carcinoma [Mesh Terms]) AND “carcinoma” [Mesh Terms] OR “endometrial cancer” [Title/Abstract]). The reference lists of relative articles were also screened to further identify potential studies.

### 2.4. Criteria for Selecting Data

We selected data with the following criteria to be included in this study: (1) the data include both case group and control samples, (2) the data is published together with some paper with full text, (3) standard methods like IHC were accompanied with the diagnosis of EC, (4) the amount and information of data were enough for an accurate evaluation on the hazard ratio for survival with 95% CI, and (5) RUNX3 expression study was conducted on primary EC tissue (not serum or other kinds of specimen). If there are some duplicated studies, we prefer the most informative or most recent one.

### 2.5. Data Extraction

The data were extracted similar to Li et al. [23].

### 2.6. Statistical Analysis

We used Cochrane RevMan 5.3.0 (the Cochrane Collaboration, Copenhagen) to perform statistical analyses. Specifically, we use risk ratio (RR) to present dichotomous data and mean difference with 95% CI to present continuous variables. The heterogeneity of the data was tested by the Chi-square test, and a data is deemed significant if *P* < 0.1. We used *I*-square to estimate total variation. We drew a funnel plot to assess the potential publication bias and used pooled estimates of RRs and their 95% CI to compare dichotomous measures. The significance threshold was set to be *P* < 0.05.

## 3. Results

### 3.1. EC Group vs. Control Group

Five studies [17, 18, 20–22] reported low RUNX3 expression in the EC group (EC tissues) and control group (normal gastric tissues). Meta-analysis via random effect model indicated that the expression rate of RUNX3 in the EC group was higher than that in the control group. The difference between the two groups was statistically significant (RR = 0.5, 95% CI (0.44, 0.57), *P* < 0.00001, Figure 2).

### 3.2. LN Metastasis of EC Tissues: Positive Group vs. Negative Group

Five studies [18–22] reported RUNX3 expression in positive and negative LN metastasis of EC tissues. Meta-analysis via random effect model showed that low RUNX3 expression rate in the positive group (LN+) was higher than that in the negative group (LN-). The difference between the two groups was not statistically significant (RR = 0.79, 95% CI (0.52, 1.19), *P* = 0.26, Figure 3).

### 3.3. TNM Stage of EC Tissues: III–IV Stage Groups vs. I–II Stage Groups

Five studies [18–22] reported the expression of RUNX3 in the II–IV stage groups and I–II stage groups of EC tissues. Meta-analysis via random effect model showed that low RUNX3 expression rate in the III–IV stages was higher than that in the I–II stage groups. The difference between the two groups was statistically significant (RR = 3.55, 95% CI (2.11, 5.98), *P* < 0.00001, Figure 4).

### 3.4. Muscular Infiltration of Endometrial Cancer: <1/2 Group vs. ≥1/2 Group

Five studies [18–22] reported low RUNX3 expression in the muscular infiltration < 1/2 group and ≥1/2 group in EC tissues. Meta-analysis via random effect model showed that low RUNX3 expression rate in the muscular infiltration of ≥1/2 group was higher than that in the <1/2 group. The difference between the two groups was statistically significant (RR = 2.38, 95% CI (1.71, 3.31), *P* < 0.00001, Figure 5).

### 3.5. Pathological Classification of Endometrial Cancer: G1 Group vs. G2–G3 Group

Five studies [18–22] reported low RUNX3 expression in the pathological classification of G1 group and G2–G3 groups in EC tissues. Meta-analysis via random effect model showed that low RUNX3 expression rate in the G1 group was higher than that in the G2–G3 groups. The difference between the two groups was statistically significant (RR = 3.19, 95% CI (2.25, 4.51), *P* < 0.00001, Figure 6).

### 3.6. Publication Bias

A funnel plot of every two groups in comparison above was applied with RR as the *x*-axis and SE (RR) as the *y*-axis. The plot was symmetric, suggesting that publication bias was minimal (Figure 7).

## 4. Discussion

The RUNX3 gene is a member of the Runt family, which includes RUNX1, RUNX2, and RUNX3. RUNX3 is located on human chromosome 1p36.1. The total length of the gene is approximately 67 kb and includes two promoters and six exons [24]. Given the high GC content of RUNX3 promoter, which accounts for approximately 64%, methylation is likely to occur [25]. RUNX3 regulates cell growth and apoptosis and exhibits important and complex transcriptional effects on cell signalling and other biological effects. The lack of RUNX3 expression is closely related to the occurrence and development of various human malignant tumours [26, 27]. RUNX3's anticancer mechanism is closely related to the TGF-*β* pathway, which functions as a growth suppressor and apoptosis-inducing factor. TGF-*β* is a growth factor that inhibits many developmental and physiological processes. A disorder of its signal pathway is involved in the occurrence and development of many tumours [18, 28]. The RUNX3 expression is abnormal in various gastrointestinal tumours, such as gastric cancer [29]. Therefore, RUNX3 is currently considered as a tumour suppressor gene. The role of RUNX3 in endometrial carcinogenesis has recently attracted increasing attention from scholars worldwide [30].

Given the biological properties of RUNX3, some scholars believe that studying the action pathway and mechanism of RUNX3 can provide new targets and insights into the treatment of uterine malignant tumours in the clinic [21]. Despite various basic and clinical studies on RUNX3 and endometrial cancer, no consensus opinion has been reached in detail. In the current study, we systematically reviewed the correlation between low expression and the clinical significance of RUNX3 in endometrial cancer. We found that low RUNX3 expression rate in the EC group is higher than that in the control group by meta-analysis. Low RUNX3 expression was not related to LN metastasis but is associated to TNM stage, degree of muscular infiltration, and pathological degree. In conclusion, low RUNX3 expression and its clinical-pathological features are closely related in endometrial cancer. RUNX3 may play a critical role in the pathophysiology, integration, and complementation of endometrial cancer. Nevertheless, the translational potentials of these findings warrant further investigation.

Although this systematic review is aimed at providing the best possible estimate of the correlation between the low expression and clinical significance of RUNX3 in endometrial cancer, it suffers from several limitations. Firstly, the number of studies and patients included in the current meta-analysis is relatively small. Secondly, all the studies were based on the Asian population, including 6, 1, and 1 from China, Korea, and Japan, respectively. Significant differences, such as those in aetiology, biological features, clinical types, and prognosis in the risk of EC, exist among various ethnic groups within a given geographical area. Given the lack of statistics on the Western population, data on the low expression rate of RUNX3 in Western patients are unavailable. Second, EC is quite heterogeneous; the sequencing of single cell RNA data of EC patients might contribute to understanding in-depth mechanisms of EC [31–34]. Finally, it will be helpful for clinical usage to identify drugs targeting EC through drug repositioning or drugs targeting this gene [35–37]. In virtue of several limitations and inconsistent combined results, further large, well-designed prospective cohort studies with good exposure assessment are warranted to confirm the findings from our study and provide further evidence.

## Figures and Tables

**Figure 1:** Flow chart for the selection of studies.

**Figure 2:** Meta-analysis of RUNX3 expression in the endometrial cancer and control group.

**Figure 3:** Meta-analysis of RUNX3 expression in LN (+) and LN (-) endometrial cancer.

**Figure 4:** Meta-analysis of low RUNX3 expression in the II–IV stage groups and I–II stage groups.

**Figure 5:** Meta-analysis of low RUNX3 expression in the muscular infiltration < 1/2 group and ≥1/2 group.

**Figure 6:** Meta-analysis of low RUNX3 expression in the G1 group and G2–G3 groups.

**Figure 7:** Funnel plot: (a) low RUNX3 expression in the EC group and control group; (b) low RUNX3 expression in the LN (+) and LN (-) EC group; (c) low RUNX3 expression in the III–IV stage groups and I–II stage groups; (d) low RUNX3 expression in the muscular infiltration of the EC < 1/2 group and ≥1/2 group; (e) low RUNX3 expression in the G1 group and G2–G3 groups in endometrial cancer.

**Table 1:** General characteristics of included studies.

Studies	Year	Country	Cases (*n*)	Age	Method	RUNX3 expression rate (%)	Group
Dong	2018	Korea	61	—	IHC	49.1%	(2) (3) (4)
Zhang	2013	China	120	—	IHC	66.6%	(1) (2) (3) (4) (5)
Liu	2013	China	117	—	IHC	73.5%	(1) (2) (3) (4) (5)
Zhang	2012	China	100	25–81	IHC	80%	(1) (2) (3) (4) (5)
Guo	2011	China	162	38–72	IHC	26.4%	(1) (2) (3) (4) (5)
He	2010	China	98	28–72	IHC	79.5%	(1) (2)
Feng	2010	China	140		IHC	42.8%	(1) (2) (3) (4) (5)
Tatsuo	2008	Japan	29		IHC	82.75	(1)

## Data Availability

The analyzed data are available from the corresponding author on reasonable request.
